The article "Large Pleural Lipoma Manifesting With Chronic Shoulder Pain" was retracted in 2024. Reasons: false authorship; unreliable results or conclusions; no approval from an author; concerns about the authorship.

# Large Pleural Lipoma Manifesting With Chronic Shoulder Pain

**DOI:** 10.7759/cureus.21113

**Published:** 2022-01-11

**Authors:** Aljawharah A Alotaibi, Fawaz S Albaqami, Asim K Almushayqih, Ghadeer N Alotaibi, Najd F Aldakkan, Jumanah M Muammar, Ahmed A Alsulaimani, Khlood I Alrowathi, Abdulwahab A Almansour, Saad S Alrushud, Alaa A Aldeibani, Amal H Allohaibi, Basmah M Aljohani, Ahmed Aljohani, Faisal Al-Hawaj

**Affiliations:** 1 Medicine, King Abdulaziz University, Jeddah, SAU; 2 Medicine, Qassim University, Qassim, SAU; 3 Medicine, Dar Al-Uloom University, Riyadh, SAU; 4 Medicine, Ibn Sina National College for Medical Studies, Jeddah, SAU; 5 Medicine, King Saud University, Riyadh, SAU; 6 Medicine, Imam Abdulrahman Bin Faisal University, Dammam, SAU

**Keywords:** lipoma, shoulder pain, musculoskeletal disorders, pleural cavity, case report

## Abstract

Musculoskeletal symptoms related to orthopedic conditions are highly prevalent worldwide and are a leading cause of morbidity. However, non-orthopedic conditions may also present with musculoskeletal symptoms. For example, shoulder pain may be caused by gastrointestinal, hepatobiliary, cardiac, and neurological pathologies. We report the case of a 32-year-old man who presented to the orthopedic clinic with a complaint of left shoulder pain for the past three months. He described the pain as sharp in nature. The pain was constant and was not related to the shoulder movements. It was not associated with morning stiffness. He had no history of preceding trauma. On examination, both shoulders were symmetrical with no evidence of deformities. Palpation over the shoulder region did not elicit any tenderness. The range of motion in both the active and passive movements was intact. The Neer and Jobe tests were negative. Also, the sensory examination was intact, and laboratory findings were normal. The patient underwent a plain frontal radiograph of the chest, which revealed a large well-circumscribed lobulated mass lesion in the left hemithorax, arising from the pleural lining. A thoracic CT scan was then performed to provide further characterization of the mass lesion and it re-demonstrated the mass as having homogeneous fat-attenuation with thin septations, probably representing pleural lipoma. The tumor was successfully resected via open thoracotomy. The patient's symptoms resolved and he had no recurrence after one year of follow-up. Pleural lipoma is a very rare benign mesenchymal tumor. The case highlights the importance of considering non-orthopedic conditions in the differential diagnosis of shoulder pain in patients with normal physical examination findings. A CT scan is vital to make the diagnosis and can show the accurate anatomic relations with respect to the tumor for surgical planning.

## Introduction

Musculoskeletal disorders are highly prevalent conditions that lead to a high economic burden on healthcare systems and societies. The Global Burden of Disease study has illustrated that musculoskeletal disorders are the leading cause of non-communicable disease disability [1]. While the majority of musculoskeletal pain cases are mechanical in nature, non-orthopedic conditions may also present with musculoskeletal symptoms. Shoulder pain is typically caused by rotator cuff injury, impingement syndrome, tendinitis, bursitis, avascular necrosis, and osteoarthrosis [2]. However, a wide variety of clinical conditions may present with referred shoulder pain. For instance, shoulder pain may result from diaphragmatic irritation that can be caused by perforated viscus, ectopic pregnancy rupture, and splenic laceration [3]. Additionally, compression of the exiting cervical nerves due to disc osteophyte complexes or spinal canal stenosis is a major cause of referred shoulder pain [3]. In such cases, careful physical examination is crucial and normal shoulder movements are a hint to consider the possibility of referred shoulder pain. In this report, we discuss the case of an otherwise healthy man presenting with chronic shoulder pain that was found to be associated with a giant pleural lipoma.

## Case presentation

A 32-year-old man presented to the orthopedic clinic with a complaint of left shoulder pain for the past three months. He described the pain as sharp in nature. The pain was constant, not related to the shoulder movements, and non-radiating. He scored it as 4/10 on the severity scale. There was no history of preceding trauma, but the patient reported that the pain had worsened after weight-lifting exercise. There had been no change in the severity of his pain and no history of pain in other joints. The pain was not associated with morning stiffness.

Apart from a history of mild intermittent asthma, the patient was generally healthy. He had no history of surgical interventions, and he was not taking any medications routinely. He was physically active and maintained a healthy lifestyle. There was no history of smoking or alcohol consumption. The family history was positive for celiac disease in all his siblings. He worked as a computer engineer.

On examination, both shoulders were symmetrical with no evidence of deformities. Palpation over the shoulder region did not elicit any tenderness. The range of motion in both the active and passive movements was intact. The Neer and Jobe tests were negative, and the sensory examination was intact. Accordingly, the findings suggested that shoulder pain could be secondary to pathologies extrinsic to the shoulder joint. Examination of the respiratory system revealed decreased air entry over the upper and middle zones of the left lung.

The patient underwent basic laboratory investigations. The findings revealed a hemoglobin level of 13.4 g/dL, leukocyte count of 8000/μL, and platelet count of 410,000/μL. The erythrocyte sedimentation rate (10.5 mm/hour) and the C-reactive protein (3.8 mg/dL) levels were within the normal range. The metabolic findings, including hepatic and renal function tests, were not deranged. No further workup was performed to rule out the autoimmune rheumatological disorder.

As an initial imaging investigation, the patient underwent a plain frontal radiograph of the chest (Figure 1). The radiograph revealed a large well-circumscribed lobulated mass lesion in the left hemithorax, arising from the pleural lining and compressing the left upper lung lobe. The mass was not associated with pleural effusion or rib destruction. A thoracic CT scan was performed to provide further characterization of the mass lesion (Figure 2). It re-demonstrated the mass as having homogeneous fat-attenuation with thin septations and arising from the chest wall pleura. These findings were suggestive of pleural lipoma.

**Figure 1:** Plain frontal chest radiograph demonstrating left opacity making an obtuse angle with the pleura suggestive of pleural tumor

**Figure 2:** Axial (A) and sagittal (B) CT images show fat-density tumor with thin septation arising from the pleural lining suggestive of pleural lipoma CT: computed tomography

Given the large size of the tumor and the patient’s symptoms, he was prepared for the surgical removal of the mass. He was referred to a tertiary center with thoracic surgery facilities. An open left thoracotomy was performed, which revealed a smooth surface tumor arising from the pleura and occupying most of the left thoracic cavity. There was no evidence of invasion of surrounding structures. The entire mass lesion was successfully removed. The diagnosis was confirmed to be pleural lipoma with no evidence of malignant sarcomatous changes. The operation and the recovery were not remarkable for any complications.

The patient had his follow-up in the family medicine clinics. He reported significant improvement in his symptoms following the surgery. After one year of regular follow-up, no active issues were reported by the patient to suggest any disease recurrence.

## Discussion

We reported a case of a large pleural lipoma manifesting as left shoulder pain. Lipoma is a benign soft tissue tumor arising from mature adipose cells. It can virtually develop in any region of the body. The thoracic cavity is among the uncommon sites for lipoma lesions. In particular, pleural lipoma is exceedingly rare [4].

Considering their slow growth and benign nature, these tumors become symptomatic when they reach a significant size and cause mass effect [5]. In our case, because of its apical location, it manifested with shoulder pain owing to the possible compression effect on the brachial plexus. It was interesting that the patient reported no history of shortness of breath despite the large size of the tumor. Pleural lipomas may even result in cardiac arrest due to the direct compression on the heart [6].

Pleural lipoma is often detected incidentally on plain chest radiographs. However, a CT scan is the method of choice to provide a detailed assessment of the lesion and surgical planning [5]. The mass lesion typically has homogeneous fat attenuation [4]. In the present case, the mass had thin septations seen in the CT scan.

The management of pleural lipoma depends on its size and clinical findings [5]. In our case, given the large size and the symptomatic nature of the tumor, surgical resection was performed. For small pleural lipomas, clinical observation with serial plain radiographs may be advised [5]. The surgical resection can be performed by conventional open thoracotomy or by video-assisted thoracoscopy [4]. However, thoracoscopy may not be feasible for large-sized tumors, as in the present case. The prognosis of intrathoracic outcomes is generally excellent. Recurrence is uncommon and is probably related to incomplete resection rather than true recurrence [4].

## Conclusions

Pleural lipoma is a very rare benign mesenchymal tumor. Our case highlights the importance of considering non-orthopedic differential diagnoses of shoulder pain in patients with normal physical examination findings. A CT scan is crucial for the diagnosis and illustrates the accurate anatomic relations with respect to the tumor for surgical planning. The prognosis of the tumor is good with a low recurrence rate if the tumor is completely resected.
